# Environmental and Genetic Factors in the Pathogenesis of COPD in the Road-Working Population

**DOI:** 10.1155/2021/9953234

**Published:** 2021-04-29

**Authors:** Yumin Zhou, Man Wang, Weiyan Yang, Jianjun Li, Jialin Li, Yueying Hu, Wei Wang, Chunli Che, Hong Qi

**Affiliations:** ^1^State Key Laboratory of Respiratory Disease, National Center for Respiratory Diseases, Guangzhou Institute of Respiratory Diseases, The First Affiliated Hospital of Guangzhou Medical University, Guangzhou 510120, China; ^2^Harbin Medical University, Harbin 150010, China; ^3^Department of Respiratory Medicine, Southern University of Science & Technology Hospital, Shenzhen 518012, China; ^4^State Key Laboratory of Urban Water Resource and Environment, Harbin Institute of Technology, Harbin 150090, China

## Abstract

**Background:**

Chronic obstructive pulmonary disease (COPD) is a typical heterogeneous condition caused by environmental and genetic risk factors.

**Objectives:**

We investigated extrinsic (environmental) and intrinsic (genetic) factors contributing to the development of COPD in a nonsmoker road-working population in Northeast China.

**Method:**

The target population was divided into a COPD group and an exposed control group. Another healthy nonroad working nonsmoker control group was also included for environmental factor comparison. Peripheral blood was collected and analyzed using inductively coupled plasma mass spectrometry for inorganic elements of PM2.5, and microarray, rt-PCR, and Multiplex ELISA for genetic factors.

**Results:**

Forty-three COPD road workers, thirty-nine non-COPD road workers, and 52 age and gender-matched healthy nonroad workers were enrolled. There were significantly higher levels in all 24 inorganic elements in the COPD group compared with the healthy control group except potassium and manganese, while the majority of inorganic elements were similar between the COPD group and the exposed control group except in aluminum and cobalt. There were 39 genes showing significant differences between the COPD group and the exposed control group. Collagen, type XV, alpha 1 (COL15A1), Meis homeobox 1 (MEIS1), carbonyl reductase 3 (CBR3), and amine oxidase, copper containing 3 (AOC3) were confirmed by rt-PCR to be differentially expressed. Their correlations with blood cytokines were also evaluated.

**Conclusions:**

Aluminum might contribute to the development of COPD in the road-working population. CBR3 and AOC3 seem expressed in different patterns than previously reported, evidenced by their correlation with proinflammatory and anti-inflammatory cytokines.

## 1. Introduction

Chronic obstructive pulmonary disease (COPD) is characterized by exacerbation episodes and is frequently associated with comorbid conditions [1]. The incidence, prevalence, and mortality rates of COPD remain high [2]; therefore, it is very important to identify the causes and pathogenesis of COPD. It is now clear that COPD is a typical heterogeneous condition [3]. The development and acute exacerbation of COPD are related to the short-term heavy exposure and/or long-term chronic exposure of atmospheric fine particulate matter (PM2.5) [4, 5]. We have shown that in COPD patients, the levels of components of PM2.5 in the bronchoalveolar lavage fluid (BALF) are higher than those in the blood [6]. However, it is still unclear which components of PM2.5 in the blood contribute to the pathogenesis of COPD.

Inorganic components have always been considered as the main pollutants in toxic PM, which are stable in nature, slower to decompose in the body, and the detection methods are more accurate [7]. Although our previous study detected PM2.5 in the BALF of COPD patients [6], the detection of PM2.5 component in blood samples, considering its easy access and as a confirmation of direct accumulation of PM2.5 in blood, is still rarely reported. In this study, we investigated intrinsic (genes) and extrinsic (environmental) factors contributing to the development and exacerbation of COPD in a road-working traffic police population in Northeast China.

## 2. Materials and Methods

All experimental protocols in this study were approved by the Institutional Ethics Committee of the First Affiliated Hospital of Harbin Medical University, and all procedures involving human were carried out in accordance with the World Medical Association Declaration of Helsinki. Written informed consent was obtained from enrolled participants.

### 2.1. Sample Collection

The target population was road-working traffic police in the region who received physical examination in October 2019. Healthy volunteers engaged in nonoutdoor work who received physical examination and agreed to participate at the same time were enrolled as healthy controls (group C). The road-working participants were divided into a COPD study group (group A, the traffic police population diagnosed as COPD) and an exposed control group (group B, the traffic police population not diagnosed as COPD). Participants in groups A and B met all the following criteria: (1) continuous work as traffic police on the road for more than 5 years; (2) nonsmoking (smoking was defined as >400 cigar/year, and >1 year before the time of physical exam); (3) aged over 30 years old; and (4) no other complicated diseases, such as infection, cancer, endocrine disease, and hypertension. COPD was diagnosed according to the 2019 GOLD criteria [8]. Five ml of fasting peripheral blood samples was collected during physical examination, aliquoted, and stored in a -80°C freezer before analyses.

### 2.2. Determination of Inorganic Elements of PM2.5 in Blood Samples

Inorganic elements in blood samples were determined as described before [6]. Briefly, 0.5 ml of blood sample was transferred into a colorimetric tube incubated with 10% nitric acid and, sequentially, added with 1 ml of concentrated nitric acid (MOS grade), 0.5 ml of 30% hydrogen peroxide of MOS grade, and digested in water bath at 100°C for 3 h, followed by addition of 2% nitric acid of MOS grade for a total volume of 2 ml. The prepared sample was filtered, transferred to a 5 ml disposable centrifugal tube, and analyzed in an inductively coupled plasma mass spectrometry (ICP-MS, Thermo Fisher Inc., US) according to the manufacturer's manual [9].

### 2.3. Microarray Analysis

Half ml of blood sample from each participant in the COPD group was randomized into three subgroups (*n* = 14, 14, and 15, respectively) and, similarly, subgrouped in the exposed control group (*n* = 13, 13, and 13, respectively). Blood samples in each subgroup were mixed together and treated with Trizol (Invitrogen) for total RNA extraction, which was quantified using NanoDrop-2000 (Thermo Scientific), and the integrity was checked by Agilent Bioanalyzer 2100 (Agilent Technologies). QIAGEN RNeasy Kit was used to further purify total RNA, out of which 250 ng was used for microarray using a human Gene expression chip (LC Biotech Human lncRNA Microarray 4 × 180 K) [10, 11]. Chips were then scanned on an Agilent Scanner G5761A (Agilent Technologies), and images were analyzed with the Feature Extraction software version 12.0.3.1 (Agilent Technologies) using default parameters. Raw data were normalized in a quantile algorithm with Genespring version 14.8 (Agilent Technologies). Genes with a *P* value < 0.05 between the exposed COPD group and the exposed control group using *t*-test were candidates for Gene Ontology (GO) and Kyoto Encyclopedia of Genes and Genomes (KEGG) analyses for biological function and pathway analysis.

### 2.4. qRT-PCR Verification of Genes

One ml of blood sample from each participant was treated with Trizol (Invitrogen) for RNA extraction, and 50 ng of the extracted total RNA was reverse transcribed into cDNA using a reverse transcriptase cDNA synthesis kit (Toyobo, Osaka, Japan), and qPCR was performed using an Entrans 2X qPCR Probe Master Mix (ABclonal) in a CFX96 Real-Time System (BIO-RAD) according to the manufacturer's manual. Comparative quantification was assessed based on the 2^−*Δ*Ct^ method using *β*-actin as control. Primers are listed in Supplementary Table 1.

### 2.5. Multiplex ELISA

Serum cytokine levels were measured using the Milliplex Luminex Magpix high-sensitivity immunoassay (EMD Millipore, Burlington, MA) with the human Cytokine Autoantibody panel and analyzed using Milliplex Analyst (Millipore) [12].

### 2.6. Statistical Analysis

Categorical variables are presented as *n* (%), and continuous variables as the mean ± SD. Student's *t*-test or Fisher's exact probability test were used to compare differences between the COPD group and the exposed control group or the healthy control group. Pearson correlation coefficient was calculated to show the correlation between genes and cytokines, where a coefficient above 0.7 or below -0.7 was considered as having a strong positive or negative correlation, respectively [13]. All statistical analyses were performed using SPSS 26.0 (Chicago, IL, USA). A two-tailed *P* < 0.05 was considered to be statistically significant.

## 3. Results

There were 309 traffic police who received annual physical exam at the outpatient department of our hospital, out of which 82 participants met the inclusion criteria. Forty-three were diagnosed with COPD (group A), and 39 were without (group B). Another 52 age and gender-matched healthy nonsmokers (determined by annual physical exam) who received annual physical exam and had careers unrelated to outdoor working, mining, chemical industry, or professional driver were selected as healthy controls (group C). The characteristics were shown in Table 1.

### 3.1. Inorganic Components of PM2.5 in Peripheral Blood

There were significantly higher levels in all 24 inorganic elements in the COPD group compared with the healthy control group except potassium and manganese, while the majority of inorganic elements were similar between the COPD group and the exposed control group except in aluminum and cobalt (Table 2), with aluminum above normal blood level.

### 3.2. Different Gene Expression in Peripheral Blood of COPD Patients by Microarray

The top 200 most differentially expressed genes between the COPD group and the exposed control group were shown in Figures 1(a)–1(d), and the involved pathways were also presented. There were 39 genes showing significant difference between the COPD group and the exposed control group (*P* < 0.05, Table 3).

### 3.3. Genes Validated by Rt-PCR

Out of the 39 genes, we found through KEGG analysis that collagen, type XV, alpha 1 (COL15A1), Meis homeobox 1 (MEIS1), carbonyl reductase 3 (CBR3), and amine oxidase, copper containing 3 (AOC3) could be candidates involved in the development of or exacerbation of COPD. We then did rt-PCR using *β*-actin as an internal control and confirmed that the first 3 genes were significantly upregulated and AOC3 was significantly downregulated in the COPD group compared with those of the exposed control group (Figure 1(e)).

### 3.4. Analysis of Different Cytokine Levels in Peripheral Blood of COPD Patients

Serum cytokine levels were measured using ELISA-based Multiplex, and the correlation between the 39 genes and 16 cytokines was shown in Figure 2. Using a coefficient above 0.7 or below -0.7 as thresholds for strong correlation, COL15A1 was positively correlated with proinflammatory cytokines IL-2 (*r* = 0.86), IL-5 (*r* = 0.88), and IFN-*γ* (*r* = 0.74), and conditional proinflammatory cytokine IL-6 (*r* = 0.88), while negatively correlated with proinflammatory cytokine IL-1*α* (*r* = −0.71). MEIS1 was positively correlated with proinflammatory cytokines IL-2 (*r* = 0.85), IL-5 (*r* = 0.79), TNF-*β* (*r* = 0.80), and IFN-*γ* (*r* = 0.97); conditional proinflammatory cytokine IL-6 (*r* = 0.71); and anti-inflammatory cytokine IL-10 (*r* = 0.71). CBR3 was positively correlated with proinflammatory cytokines IL-2 (*r* = 0.78), TNF-*β* (*r* = 0.70), and IFN-*γ* (*r* = 0.71). AOC3 was negatively correlated with proinflammatory cytokines IL-2 (*r* = −0.70), IL-12p40 (*r* = −0.73), TNF-*β* (*r* = −0.71), and IFN-*γ* (*r* = −0.73).

## 4. Discussion/Conclusion

Aluminum has been reported to be involved in the development of COPD [14]. In our study, there was a significantly higher level of aluminum in the blood of COPD patients compared with that of the exposed controls, suggesting that the blood level of aluminum could be a cause leading to COPD. Some studies have shown that certain components in PM2.5, such as metals and polycyclic aromatic hydrocarbons, stimulate the release of reactive oxygen species (ROS) from lung epithelial cells, which can damage cilia, increase mucus production, block airway, and lead to difficulty in breathing [15, 16].

The inflammatory response is one of the important pathogenesis of COPD. With the development of high-throughput sequencing technology, PM2.5 has been shown to affect the expression of genes. In bronchial epithelial cells collected from COPD patients, maternally expressed gene 3 (Meg3), a long noncoding RNA, is upregulated after exposure to fine PM and is negatively correlated with FEV1% [17]. It has been reported that PM2.5 can inhibit RhoA activity by overactivating PI3K*δ*, causing abnormal cytoskeletal rearrangement, weakening the defective phagocytic ability of alveolar macrophages, and aggravating oxidative stress in mice with COPD [18]. Li et al. showed that after healthy young people were exposed to PM2.5 for a short period of time, genes regulating inflammation and oxidative stress were methylated [19]. The triple motif methylation of 45 (TRIM45) gene is significantly higher under high PM2.5 exposure. The target protein of this gene regulates the MAPK and NF-*κ*B signaling pathways, which play an important role in the inflammatory response [20]. Therefore, exposure to atmospheric fine particles may affect the expression of COPD genes, and abnormal gene expression will also affect COPD, forming a vicious circle that affects the progress of COPD.

Through microarray analysis, we found 39 differentially expressed genes between the COPD and exposed control groups. Among the four rt-PCR validated genes, COL15A1 is involved in protein digestion and absorption and is identified in asthma-idiopathic pulmonary fibrosis [21]. MEIS1 is involved in signaling pathways regulating pluripotency of stem cells as well as transcriptional misregulation in cancers and is hypermethylated in COPD smokers [22]. CBR3 is involved in the metabolism of arachidonic acid and xenobiotics by cytochrome P450 and is highly expressed in Keap knockout mice that protected Clara cells against oxidative stress ex vivo and attenuated oxidative stress and cigarette smoke-induced inflammation in vivo [23]. AOC3 is involved in the metabolism of glycine, serine, threonine, tyrosine, phenylalanine, and beta-alanine, as well as in leukocyte recirculation by oxidizes primary amines to produce hydrogen peroxide, aldehyde, and ammonia, contributing to leukocyte adhesion [24]. Thus, the increase in CBR3 and decrease of AOC3 at RNA level in the COPD group participants in our study hinted their extra roles in COPD and need further validation by proteomic studies.

Serum cytokines are involved in the development of nonsmoking COPD after exposure to PM2.5 [25]. Major anti-inflammatory cytokines include IL-4, IL-10, and IL-13, whereas IL-6 is either anti-inflammatory or proinflammatory, under various conditions [26–28]. In the COPD participants in our study, CBR3 was positively correlated with proinflammatory cytokines, and AOC3 was negatively correlated with proinflammatory cytokines, which are consistent with their differentiated expression level. Although none of the participants in the present study received influenza and pneumonia vaccines during their annual physical exam, it is still interesting to note that those vaccines might not be associated with COPD [29]. Single-nucleotide polymorphisms [30, 31] and ambient PM2.5-bound organic and inorganic chemicals [32] might also be involved in the pathogenesis of COPD that warrants further investigations.

In conclusion, we found that aluminum might contribute to the development of COPD in the road-working population. CBR3 and AOC3 seem expressed in different pattern than previously reported, supported by their correlation with cytokines. Our findings provided novel insights into future studies in the development of COPD.

## Figures and Tables

**Figure 1:** Microarray analysis. (a) Heatmap of sequencing result (top 200 genes). Red: increased gene level; green: decreased gene level. (b) Volcano plot of microarray results. (Blue dots were significantly decreased genes, while red dots were significantly increased genes, *P* < 0.05, respectively). (c) Bar plot of GO analysis. (d) ggplot of KEGG analysis. (e) Validation of gene expression by rt-PCR. Blue bars represent exposure control, and orange bars represent COPD cases (*n* = 35 in each group, *P* < 0.05 in all comparisons).

**Figure 2:** Correlation between 39 genes and 16 cytokines in COPD cases by Pearson correlation coefficient (*n* = 43). On the top, anti-inflammatory cytokines were labeled in orange, while conditional anti-inflammatory cytokines were in green.

**Table 1:** Characteristics of enrolled participants.

	Group A (43 total)	Group B (39 total)	Group C (52 total)	*P* value (A vs. B)	*P* value (A vs. C)
Age	47.2 ± 8.8	49.1 ± 8.0	46.9 ± 8.2	0.31	0.86
Gender (male)	40	35	43	0.60	0.13
Years of road work	14 ± 5.9	13 ± 5.1	—	0.42	—

**Table 2:** Inorganic component of PM2.5 in the blood of participants by ICP-MS tests.

Elements	Normal range	Measured blood elements value					No. of participants above normal range (%)				
		Group A (*n* = 43)	Group B (*n* = 39)	Group C (*n* = 52)	*P* (A vs. B)	*P* (A vs. C)	Group A (*n* = 43)	Group B (*n* = 39)	Group C (*n* = 52)	*P* (A vs. B)	*P* (A vs. C)
K (mg/mL)	3.50-5.30	3.80 ± 0.36	3.74 ± 0.33	3.77 ± 0.35	0.44	0.68	0	0	0	1	1
Al (*μ*g/mL)	0.005-0.465	4.19 ± 0.33	3.85 ± 0.28	0.0027 ± 0.002	**<0.001**	<0.001	43 (100)	39 (100)	6 (11.54)	1	<0.001
Mg (*μ*g/mL)	3.31-5.02	4.34 ± 1.56	4.32 ± 1.45	3.17 ± 1.54	0.95	<0.001	10 (23.26)	0	1 (1.92)	**0.001**	<0.01
Fe (mg/mL)	3.72 -6.46	4.49 ± 0.85	4.70 ± 0.69	3.07 ± 1.19	0.23	<0.001	0	0	0	1	1
Ca (*μ*g/mL)	4.57-7.58	8.21 ± 5.81	7.79 ± 3.83	6.01 ± 2.68	0.70	0.02	25 (58.14)	15 (38.46)	3 (5.77)	0.07	<0.001
Pb (*μ*g/mL)	0.0225-0.13	2.53 ± 2.98	2.49 ± 2.45	0.13 ± 0.11	0.94	<0.001	43 (100)	39 (100)	10 (19.23)	1	<0.001
Zn (ug/mL)	6.32-22.57	11.57 ± 7.88	11.30 ± 6.98	8.40 ± 3.29	0.87	<0.01	5 (11.62)	6 (15.38)	1 (1.92)	0.62	0.09
Ba (*μ*g/mL)	0.002-0.218	0.49 ± 0.55	0.39 ± 0.35	0.15 ± 0.15	0.33	<0.001	43 (100)	26 (66.67)	5 (9.61)	**<0.001**	<0.001
Cu (*μ*g/mL)	0.66-1.05	0.92 ± 0.26	0.91 ± 0.18	0.30 ± 0.02	0.84	<0.001	10 (23.26)	6 (15.38)	0	0.37	<0.001
Cr (*μ*g/mL)	0.003-0.025	1.088 ± 0.8	0.89 ± 0.63	0.04 ± 0.01	0.22	<0.001	43 (100)	39 (100)	52 (100)	1	1
Ti (*μ*g/mL)	0.105-0.292	4.32 ± 3.26	3.88 ± 3.03	0.032 ± 0.039	0.53	<0.001	43 (100)	39 (100)	0	1	<0.001
Mn (*μ*g/mL)	0.008 -0.028	0.187 ± 0.35	0.13 ± 0.08	0.102 ± 0.04	0.32	0.09	43 (100)	39 (100)	6 (11.54)	1	<0.001
Rb (*μ*g/mL)	2.12-4.46	2.45 ± 0.56	2.58 ± 0.48	2.51 ± 0.65	0.26	0.48	0	0	0	1	1
Cd (*μ*g/mL)	0.0007-0.002	0.067 ± 0.08	0.069 ± 0.06	0.009 ± 0.02	0.90	<0.001	43 (100)	39 (100)	14 (26.92)	1	<0.001
Sr (*μ*g/mL)	0.012-0.05	0.076 ± 0.04	0.072 ± 0.036	0.014 ± 0.037	0.64	<0.001	21 (48.83)	23 (58.85)	2 (3.85)	0.36	<0.001
Ni (*μ*g/mL)	0.009-0.036	0.081 ± 0.074	0.062 ± 0.048	0.004 ± 0.005	0.18	<0.001	30 (69.76)	28 (71.79)	1 (1.92)	0.97	<0.001
V (*μ*g/mL)	0.0006-0.005	0.056 ± 0.05	0.046 ± 0.04	0.001 ± 0.0006	0.32	<0.001	43 (100)	39 (100)	0	1	<0.001
Ag (*μ*g/mL)	0.00005-0.002	0.009 ± 0.02	0.006 ± 0.007	0.0017 ± 0.001	0.38	0.01	43 (100)	39 (100)	13 (25)	1	<0.001
Se (*μ*g/mL)	0.171-0.310	0.129 ± 0.12	0.110 ± 0.02	0.0008 ± 0.001	0.33	<0.001	1 (2.32)	0	0	1	0.45
Mo (*μ*g/mL)	0.0005-0.004	0.008 ± 0.008	0.006 ± 0.006	0.0008 ± 0.001	0.21	<0.001	5 (11.62)	3 (7.69)	3 (5.77)	0.72	0.46
Co (*μ*g/mL)	0.005-0.89	0.003 ± 0.002	0.002 ± 0.001	0.0002 ± 0.0001	**<0.01**	<0.001	0	0	0	1	1
Sb (*μ*g/mL)	0.01-29.5	0.013 ± 0.007	0.013 ± 0.006	0.0002 ± 0.0001	1	<0.001	1 (2.32)	0	0	1	0.45
Tl (*μ*g/mL)	0.001-0.50	0.001 ± 0.007	0.001 ± 0.001	0.02 ± 0.014	1	<0.001	0	0	0	1	1
As (*μ*g/mL)	0.002-0.017	0.132 ± 0.10	0.109 ± 0.06	0.006 ± 0.006	0.22	<0.001	43 (100)	39 (100)	6 (11.54)	1	<0.001

**Table 3:** Genes showing significant changes between the COPD group and the exposure control group by microarray analysis.

Gene name	Average fold change^∗^	SD	*P* value
ESD	5.04	1.68	2.79E-02
PRKRIR	4.60	1.67	1.90E-03
RAB3IP	3.62	1.68	3.50E-03
ARHGAP26	3.35	1.85	1.41E-02
CBR3	3.23	1.79	4.80E-02
MEIS1	3.17	1.79	1.09E-02
CEMP1	3.08	1.87	8.00E-04
TTC13	3.08	1.80	1.25E-02
EDEM3	2.95	1.80	2.71E-02
ZNF737	2.90	1.80	2.10E-06
PCDH15	2.90	1.79	6.65E-04
CARD8	2.90	1.79	5.36E-03
ZNF799	2.87	1.85	4.91E-02
SLC35F4	2.82	1.85	1.41E-02
C8orf48	2.77	1.85	4.47E-02
TMTC2	2.68	1.84	1.65E-02
NPR3	2.68	1.84	1.04E-02
LAMA1	2.63	1.89	1.47E-02
FBXW2	2.62	1.89	7.30E-03
BCKDHB	2.62	1.89	9.00E-03
SYNE1	2.59	2.04	4.71E-02
SPEF2	2.56	2.32	2.37E-02
COL15A1	2.52	2.08	2.10E-02
CDK17	2.51	2.10	6.06E-03
ZNF461	0.45	3.43	7.22E-03
TFEC	0.45	3.45	3.68E-02
NTNG1	0.45	3.49	7.70E-03
ZNF789	0.45	3.53	1.38E-02
FAM83G	0.45	3.55	1.36E-02
SCNM1	0.44	3.25	4.41E-02
TP53I11	0.44	3.07	2.38E-02
TMEM63A	0.43	2.95	8.30E-03
AOC3	0.43	2.96	2.78E-02
HAND2	0.42	1.97	8.06E-03
ZCCHC16	0.42	1.90	8.40E-03
B3GNT4	0.41	2.05	1.10E-02
FBXO25	0.37	2.12	1.80E-03
C1orf220	0.35	2.32	1.13E-02
OFD1	0.24	3.83	1.37E-02

^∗^Compared with the exposed control group.

## Data Availability

After publication, the data will be made available to others on reasonable requests to the corresponding author. Availability of data and material also need to be approved by the Institutional Ethics Committee of the First Affiliated Hospital of Harbin Medical University.

## Additional Points

*What is Already Known about This Subject?* Chronic obstructive pulmonary disease (COPD) is a typical heterogeneous condition caused by environmental and genetic risk factors. *What Are the New Findings?* For the first time, inorganic components of PM2.5 are measured in peripheral blood. Environmental factors, such as PM2.5, and genetic factors, such as COL15A1, MEIS1, CBR3, and AOC3 genes, are involved in COPD. *How Might This Impact on Policy or Clinical Practice in the Foreseeable Future?* Regular physical examination with blood test of inorganic components of PM2.5 and occupational disease protection measures are needed in road-working population.

## Supplementary Materials

Supplementary Materials Sequence of primers for rt-PCR is listed in Table S1.

## References

[1] Vogelmeier C. F., Criner G. J., Martinez F. J. (2017). Global strategy for the diagnosis, management, and prevention of chronic obstructive lung disease 2017 report. GOLD executive summary. *American Journal of Respiratory and Critical Care Medicine*.

[2] (2018). Chronic obstructive pulmonary disease. https://www.cdc.gov/copd/data.html.

[3] Rennard S. I. (2011). COPD heterogeneity: what this will mean in practice. *Respiratory Care*.

[4] Chen R., Yin P., Meng X. (2017). Fine Particulate Air Pollution and Daily Mortality. A Nationwide Analysis in 272 Chinese Cities. *American Journal of Respiratory and Critical Care Medicine*.

[5] Wang M., Aaron C. P., Madrigano J. (2019). Association between long-term exposure to ambient air pollution and change in quantitatively assessed emphysema and lung function. *JAMA*.

[6] Che C., Li J., Dong F. (2020). Seasonal characteristic composition of inorganic elements and polycyclic aromatic hydrocarbons in atmospheric fine particulate matter and bronchoalveolar lavage fluid of COPD patients in Northeast China. *Respiratory Medicine*.

[7] Jia Y. Y., Wang Q., Liu T. (2017). Toxicity research of PM2.5 compositions in vitro. *International Journal of Environmental Research and Public Health*.

[8] Global initiative for chronic obstructive lung disease. https://goldcopd.org/wp-content/uploads/2018/11/GOLD-2019-v1.7-FINAL-14Nov2018-WMS.pdf.

[9] Cantlay T., Bain D. J., Curet J. (2020). Determining conventional and unconventional oil and gas well brines in natural sample II: cation analyses with ICP-MS and ICP-OES. *Journal of Environmental Science and Health. Part A, Toxic/Hazardous Substances & Environmental Engineering*.

[10] Ni C., Fang Q., Chen W. (2020). Breast cancer-derived exosomes transmit lncRNA SNHG16 to induce CD73+*γδ*1 Treg cells. *Signal Transduction and Targeted Therapy*.

[11] Guo Q., Wang J., Sun R. (2020). Identification of circulating hub long noncoding RNAs associated with hypertrophic cardiomyopathy using weighted correlation network analysis. *Molecular Medicine Reports*.

[12] Gordon K. B., Armstrong A. W., Foley P. (2019). Guselkumab efficacy after withdrawal is associated with suppression of serum IL-23-regulated IL-17 and IL-22 in psoriasis: VOYAGE 2 study. *Journal of Investigative Dermatology*.

[13] Mukaka M. M. (2012). Statistics corner: a guide to appropriate use of correlation coefficient in medical research. *Malawi Medical Journal*.

[14] Blanc P. D., Annesi-Maesano I., Balmes J. R. (2019). The occupational burden of nonmalignant respiratory diseases. An official American Thoracic Society and European Respiratory Society statement. *American Journal of Respiratory and Critical Care Medicine*.

[15] Figliuzzi M., Tironi M., Longaretti L. (2020). Copper-dependent biological effects of particulate matter produced by brake systems on lung alveolar cells. *Archives of Toxicology*.

[16] Xia R., Fang N., Yang Y., Xu F., Zhang L., Ji S. (2020). PM2.5 promotes apoptosis of alveolar epithelial cells via targeting ROS/p38 signaling pathway and thus leads to emphysema in mice. *Minerva Medica*.

[17] Song B., Ye L., Wu S., Jing Z. (2020). Long non-coding RNA MEG3 regulates CSE-induced apoptosis and inflammation via regulating miR-218 in 16HBE cells. *Biochemical and Biophysical Research Communications*.

[18] Xu Z., Ding W., Deng X. (2019). PM 2.5, fine particulate matter: a novel player in the epithelial-mesenchymal transition?. *Frontiers in Physiology*.

[19] Li H., Chen R., Cai J., Cui X., Huang N., Kan H. (2018). Short-term exposure to fine particulate air pollution and genome-wide DNA methylation: a randomized, double-blind, crossover trial. *Environment International*.

[20] Shibata M., Sato T., Nukiwa R., Ariga T., Hatakeyama S. (2012). TRIM45 negatively regulates NF-*κ*B-mediated transcription and suppresses cell proliferation. *Biochemical and Biophysical Research Communications*.

[21] Maghsoudloo M., Azimzadeh Jamalkandi S., Najafi A., Masoudi-Nejad A. (2020). Identification of biomarkers in common chronic lung diseases by co-expression networks and drug-target interactions analysis. *Molecular Medicine*.

[22] Staudt M. R., Buro-Auriemma L. J., Walters M. S. (2014). Airway basal stem/progenitor cells have diminished capacity to regenerate airway epithelium in chronic obstructive pulmonary disease. *American Journal of Respiratory and Critical Care Medicine*.

[23] Blake D. J., Singh A., Kombairaju P. (2010). Deletion of Keap1 in the lung attenuates acute cigarette smoke–induced oxidative stress and inflammation. *American Journal of Respiratory Cell and Molecular Biology*.

[24] Dunkel J., Aguilar-Pimentel J. A., Ollert M. (2014). Endothelial amine oxidase AOC3 transiently contributes to adaptive immune responses in the airways. *European Journal of Immunology*.

[25] Audi C., Baïz N., Maesano C. N. (2017). Serum cytokine levels related to exposure to volatile organic compounds and PM(2.5) in dwellings and workplaces in French farmers–a mechanism to explain nonsmoking COPD. *International Journal of Chronic Obstructive Pulmonary Disease*.

[26] Zhang J., An J. (2007). Cytokines, inflammation and pain. *International Anesthesiology Clinics*.

[27] Song W., Wang Y., Tian F. (2021). Clinical significance of procalcitonin, C-reactive protein, and interleukin-6 in helping guide the antibiotic use for patients with acute exacerbations of chronic obstructive pulmonary disease. *Disease Markers*.

[28] Mocan M., Mocan Hognogi L. D., Anton F. P. (2019). Biomarkers of inflammation in left ventricular diastolic dysfunction. *Disease Markers*.

[29] Bazargan M., Wisseh C., Adinkrah E. (2020). Influenza vaccination among underserved African-American older adults. *BioMed Research International*.

[30] Yu S., Xue M., Yan Z., Song B., Hong H., Gao X. (2021). Correlation between TNF-*α* -308 and +489 Gene Polymorphism and Acute Exacerbation of Chronic Obstructive Pulmonary Diseases. *BioMed Research International*.

[31] Liu Y., Huang K., Wang Y. (2020). Integration of SNP disease association, eQTL, and enrichment analyses to identify risk SNPs and susceptibility genes in chronic obstructive pulmonary disease. *BioMed Research International*.

[32] Kang Z., Liu X., Yang C., Wang C., Miao X., Na X. (2019). Effect of ambient PM2.5-bound BbFA and DahA on small airway dysfunction of primary schoolchildren in Northeast China. *BioMed Research International*.

